# Epidermal and dermal hydration in relation to skin color parameters

**DOI:** 10.1111/srt.70028

**Published:** 2024-08-21

**Authors:** Harvey N. Mayrovitz, Kawaiola Aoki, Emily Deehan, Marissa Ruppe

**Affiliations:** ^1^ Dr. Kiran C. Patel College of Allopathic Medicine Nova Southeastern University Fort Lauderdale USA; ^2^ Dr. Kiran C. Patel College of Osteopathic Medicine Nova Southeastern University Fort Lauderdale USA

**Keywords:** dermal water, erythema, Fitzpatrick skin type, gender differences, melanin, personalized skincare, skin color, skin hydration, TDC, tissue dielectric constant

## Abstract

**Background:**

Our goal was to investigate linkages between skin color parameters and skin hydration. Since most prior studies focused on stratum corneum hydration, we focused on epidermal and dermal hydration in relation to skin color parameters in both sexes.

**Materials and Methods:**

Thirty adults (16 female) with an age ± SD of 24.3 ± 0.6 years participated. Three sites on both volar forearms were evaluated for melanin index (MI), erythema index (EI), Individual Typology Angle (ITA), tissue dielectric constant (TDC) values to depths of 0.5 mm (TDC_0.5_) and 2.5 mm (TDC_2.5_), and Fitzpatrick skin type (FST).

**Results:**

MI and EI were highly correlated (*r* = 0.800, *p* < 0.001) with maximum differences in MI and ITA along the arm of 3% and 6.3% with no difference between arms. Male MI was greater than females (*p* < 0.01). Male TDC_2.5_ was 36.1 ± 5.4 and correlated with EI (*r* = 0.231, *p* = 0.035). Contrastingly, female TDC_25_ was 28.5 ± 3.6 with no correlation with EI but was correlated with MI (*r* = −0.301, *p* = 0.003). These differential patterns held true for TDC_0.5_. For both sexes, FST and ITA were highly correlated (*r* = −0.756, *p* < 0.001).

**Conclusions:**

The findings revealed several correlations between skin color parameters and hydration that differed between males in females in some cases. The observed correlations may indicate that melanin may differentially impact water‐holding capacity between sexes and provides a future research target. Further, these initial findings also may hold significance for dermatological assessments and the customization of skincare treatments tailored to individual skin types and demographics.

## 1 INTRODUCTION

Skin's hydration status is an important component of skin health,^1^ which depends on multiple factors,^2^ with its measurement widely reported using various biophysical methods,^3^ and even potentially self‐measured.^4^ Skin hydration is to be distinguished from skin's exposure to high moisture environments with associated detrimental impacts on skin integrity.^5^, ^6^ Linkages between increased skin hydration levels and firmness have been reported.^7^ This improvement may be slightly facilitated by greater water consumption,^8^ with resulting positive effects on facial wrinkles documented.^9^ In addition, skin's hydration levels have been reported to be involved in multiple processes including as a potential predictor of pressure ulcer development in at‐risk persons,^10^ as a threshold for wound healing potential in persons with diabetes mellitus,^11^ as a feature of atopic dermatitis^12^ that is improved when hydration is increased,^13^ and having a significant relationship to transcutaneous oxygen levels in patients with peripheral neuropathy.^14^ Sex‐related differences in skin hydration of the stratum corneum^15^ and dermis^16^ have also been documented. Differences in skin hydration between persons with different skin tones have been described as exemplified by lower levels of stratum corneum hydration in young African women as compared to young Caucasian women.^17^ However, the potential relationship between skin color parameters and hydration has not been systematically evaluated. The possibility of such a relationship emerges from some prior findings. A study of Japanese women exposed to larger lifetime amounts of sun‐related ultraviolet were found to have forehead skin color differences associated with reduced stratum corneum hydration.^18^ In a study that was evaluating the potential impact of adding mineral water to the diet it was noted that an increase in skin hydration was accompanied by an increase in skin surface lightness as measured by L* of the L*, a*, b* scale.^19^ Using a different skin color parameter, the Individual Typology Angle (ITA), evaluation of geriatric residents found that skin color was impacted by the nutritional status of residents but apparently not related to stratum corneum hydration.^20^ Other studies, that included facial skin features of Chinese women noted the role of skin color in perceived age and attractiveness,^21^ and the impacts of seasonal exposure,^22^ but did not relate the skin color parameters to measures of skin hydration. Other large‐scale studies of facial skin of Caucasian women that measured both stratum corneum hydration and skin color parameters indicated an age dependence.^23^ Measurements of facial skin color assessed with both L* and ITA in Korean women indicated both linearly decreased with age as did facial skin stratum corneum hydration.^24^ A comparison of hand skin dorsum L* values between Chinese and Caucasian women versus age, revealed an age‐related decrease for both with a decrease in stratum corneum hydration occurring at about age 60.^25^ A similar investigation of the age dependence of skin color parameters and skin hydration at various anatomical sites in Chinese women has been reported.^26^ However, the potential relationship between the skin color parameters and hydration levels was not specifically reported for any of the age groups evaluated. But a comparison of L* versus stratum corneum hydration measured at the upper inner arm, among Puerto Rican natives, Hispanics, Blacks and White women showed a slight but statistically significant negative association, between L* and stratum corneum hydration.^27^ Other measurements of skin color parameters and skin hydration parameters have been done to determine each's potential variations during the day, but with no attempt to investigate potential relationships reported.^28^ It was thus a specific aim of the present study to directly investigate the possible linkage between skin color and skin hydration with a focus on volar forearm skin because of its wide use in skin research and clinical evaluations for persons with upper extremity lymphedema.^29^, ^30^ The inner forearm is also less sun exposed than the face and likely represents a more natural state. Further, since most prior studies only focused on the hydration status of the upper epidermis, primarily the stratum corneum, a second aim was to measure both epidermal and dermal hydration together with their corresponding skin color parameters. In addition, since most of the prior studies have focused primarily on females as test subjects, a third aim was to include males and females and to compare their skin‐related findings with respect to skin color parameters and hydration status.

## 2 METHODS

### 2.1 Subjects

This study was approved by the Nova Southeastern Institutional Review Board (IRB, 2023‐550‐NSU). Informed consent was obtained prior to participants’ enrollment. Thirty (30) healthy adults between the age of 22–32 years volunteered to participate in this study. To participate the entry requirements were that they had no significant hair on the anterior forearm, had no known allergy to topical moisturizers, had no personal history of chronic dermatologic disease (eczema or psoriasis) or any active dermatologic disease in the area of interest (such as other allergic or infectious diseases). All participants met with one of the co‐investigators (CI) at a scheduled date and time.

### 2.2 Measurement devices

The three skin‐measuring devices used in this study were the SkinColorCatch, the MoistureMeterEpiD, and the MoistureMeterD, all manufactured by Delfin Technologies (Kuopio, Finland). The SkinColorCatch quantifies erythema, melanin, and individual typographic angle (ITA).^31^, ^32^, ^33^ The MoistureMeterEpiD measures the tissue dielectric constant (TDC) of the tissue at the epidermal level to a depth of approximately 0.5 mm,^34^, ^35^ and the MoistureMeterD that measures the TDC in the skin and subcutis to a depth of approximately 2.5 mm.^36^, ^37^, ^38^ TDC values are directly related to tissue water.^39^, ^40^, ^41^

### 2.3 Measurement procedures

While the subject was resting in a seated position, a premade template with five 1 in. diameter holes, was placed on both anterior forearms. Using a surgical grade pen, the center of each hole was marked as illustrated in Figure 1. After marking, the template was removed, and skin measurements were made adjacent to the mark on clear skin beginning on the left arm and then on the right arm at sites 1, 3 and 5 in that order along the forearm on both arms. The distance between site 1 and site 3 and between site 3 and 5 was 50.8 mm. Skin temperature was measured first followed by TDC measurement, first to a depth of 2.5 mm (TDC_2.5_) and then to a depth of 0.5 mm (TDC_0.5_). Skin temperature was measured once at each site using an infrared thermometer (Exergen, Watertown Main, USA, Model DX501‐RS)) with a stated repeatability of ± 0.1°C. Room temperature (TRM) and relative humidity (RH) were measured (Fluke Model 971, Everett, WA, USA with a stated accuracy of ± 0.1°C for TRM and ± 2.5% for RH. The Fitzpatrick score was based on the sum of the participant's rating of their genetic disposition score, their reaction to sun score and their tanning habits scores from which their skin type value (1−6) was determined.^42^

**FIGURE 1:** Measurement sites on the volar forearm. Measurements were made on non‐marked skin adjacent to the center of sites 1, 3 and 5 on the right (R) and left (L) forearms. The center‐to‐center distance between site 1 and site 3 and site 3 to site 5 are 50.8 mm. Sites 2 and 4 were not used in the present study.

### 2.4 Analysis

Analysis of possible variations in hydration parameters (TDC_2.5_ and TDC_0.5_) among forearm sites (1, 3, and 5) was assessed for the entire group (*N* = 30) using a general linear model (GLM) with forearm site as the within‐subject variable and arm as the between variable. A similar analysis was conducted to determine potential site and arm variability in skin color parameters consisting of the erythema index (EI), the melanin index (MI), and the ITA. When comparisons were made between males and females they were based on the nonparametric Mann‐Whitney test. Tests for correlations between hydration parameters and skin color parameters were done using all paired values to determine the Pearson correlation coefficient (*r*) and its significance. For the entire group (*N* = 30) there were 180 paired data points. In those cases, in which the correlations for females and males were evaluated separately, there were 96 paired values for females and 84 for males. To obtain correlations among the Fitzpatrick score, Fitzpatrick classification and ITA values, an average ITA value was used (ITA_AVG_) that was calculated for each subject as the average of the six forearm site ITA values. All statistics were done using SPSS version 16.

## 3 RESULTS

### 3.1 Subject demographics and average skin parameter values

Thirty young healthy adults (16 female) with an age range of 22 to 27 years (average age ± SD of 24.3 ± 1.6 years), were evaluated. Subject's body mass index (BMI) ranged from 17.8 to 37.1 Kg/m^2^ with an average of 24.5 ± 4.9 Kg/m^2^. Of the 30 subjects, two males and one female would be classified as obese (BMI > 30 Kg/m^2^), nine subjects would be classified as overweight (BMI > 25 Kg/m^2^), six of whom were females, and one female would be classified as underweight (BMI < 18.5 Kg/m^2^). The remainder (17 subjects) had a normal BMI between 18.5 to 24.9 Kg/m^2^. Statistically significant differences between females and males are noted in Table 1. Height and weight were greater for males but there was no gender difference in BMI. The skin average values of all measured parameters were greater in males except for the ITA value that was significantly less in males. Since, lower ITA values indicate darker skin tones, the male subjects on average had darker skin tones as a group.

**TABLE 1:** Gender comparisons of demographic and average skin color and TDC values.

	Female	Male	*p*‐value
N	16	14	
Age (years)	24.3 ± 1.5	24.2 ± 1.7	0.854
Height (cm)	162.4 ± 9.8	182.2 ± 4.8	<0.0001
Weight (Kg)	61.7 ± 7.4	84.9 ± 16.6	<0.0001
BMI (Kg/m^2^)	23.6 ± 4.4	25.6 ± 5.3	0.257
Fitzgerald Score	23.7 ± 5.4	27.9 ± 4.7	0.031
Fitzgerald Class	3.3 ± 0.79	4.0 ± 0.78	0.043
*Skin Average Parameters*			
Erythema Index	407.2 ± 21.0	426.1 ± 19.8	0.013
Melanin Index	568.3 ± 52.6	625.5 ± 67.4	0.007
IAT (degrees)	43.2 ± 14.3	28.2 ± 19.0	0.017
TDC Epidermis	33.5 ± 5.8	41.6 ± 9.2	0.017
TDC Dermis	28.1 ± 3.1	36.1 ± 5.0	<0.0001
Skin Temp (°C)	30.3 ± 0.9	31.1 ± 1.0	0.002

*Note*: Table entries are the mean ± SD. Parameters without indicated units are dimensionless. Skin average parameters are calculated as the average of all six measured forearm sites. *p*‐Values are based on the nonparametric Mann‐Whitney test.

With respect to self identified race/ethnicity, 4 participants identified as Asian (one female), 1 as Black (female), 2 as Hispanic (both female), 3 as Middle Eastern (one female), 7 as South East Asian (two female), and 13 as White (nine female).

### 3.2 Variations in skin color parameters among sites and between arms

The relationship between the MI and erythema index, based on all 180 measured sites (6 sites x 30 subjects) is shown in Figure 2, reveals a significant correlation between MI and EI (*r* = 0.800, *p* < 0.001). As summarized in Table 2, the skin MI varied among forearm sites on both arms. The most distal forearm site (site 1) tended to have the least melanin value (585 ± 67) compared to the most proximal site (site 5) whose average value was 601 ± 66. The percentage difference between the peripheral and proximal site was small averaging less than 3%. Along with the observed melanin variation there was a related pattern of decreasing values of ITA from peripheral to proximal sites. This percentage change was also not large (6.3%) but was greater than the difference in melanin between these sites. Although there was these variations along the forearm there was no significant difference in any of the color‐related parameters at any site between arms. A breakdown as to possible pattern differences between male and female subject is summarized in Table 3. For both sexes there is a highly significant but small overall increase in MI from the distal to the more proximal forearm sites. For males and females the average percentage difference between site 1 and site 5 was 2.1% and 3.4% respectively. At every site, melanin was greater for males than for females (*p* < 0.01). Variations among sites was even less for erythema and insignificant for females as shown in Table 3. However, females (but not males) showed a site dependency of ITA with the lowest ITA value at the most proximal site. The maximum differences among sites for ITA was 8.5%. For all forearm sites, the present female group had a greater ITA than for the male group (*p* < 0.01).

**FIGURE 2:** Melanin—Erythema Relationship. MI and EI as measured on all 180 forearm skin sites. Solid line is the linear regression with the associated equation shown in the figure. The *r* is the Pearson correlation coefficient and *p* is the significance of the correlation. EI, erythema index; MI, Melanin index.

**TABLE 2:** Skin color parameters by forearm site and arm for all 30 subjects.

	Site 1	Site 3	Site 5	*p*‐value (overall)
**Melanin Index**				
Left Arm	589 ± 69	602 ± 67	604 ± 63	0.00004
Right Arm	581 ± 67	596 ± 64	598 ± 69	<0.00001
Arms Combined	585 ± 67^a^	599 ± 65	601 ± 66	<0.00001
**Erythema Index**				
Left Arm	417 ± 30	416 ± 23	415 ± 22	0.913
Right Arm	418 ± 22	414 ± 22	415 ± 21	0.001
Arms Combined	418 ± 26	415 ± 22	415 ± 21	0.118
**Individual Typology Angle (ITA, degrees)**				
Left Arm	37.2 ± 18.6	35.9 ± 19.8	34.9 ± 17.7	0.018
Right Arm	37.1 ± 18.3	37.0 ± 17.4	35.0 ± 17.8	0.012
Arms Combined	37.2 ± 18.3	36.5 ± 18.5	35.0 ± 17.6^a^	0.0004

*Note*: Table entries are the mean ± SD. Parameters without indicated units are dimensionless. Site 1 is closest to the wrist and site 5 is closest to the cubital crease. *p*‐Values are based on a general linear model (GLM) for repeated measures with site as the within repeated measure. Significance of pairwise comparisons between sites are adjusted according to a Bonferroni correction.

^a^ Indicates sites different from the others (*p* < 0.01). No parameters significantly differed between arms.

**TABLE 3:** Male versus female skin color parameters.

	Site 1	Site 3	Site 5	*p*‐value (overall)
**Melanin**				
Male	618 ± 67^a^	628 ± 67	631 ± 66	0.00007
Female	556 ± 54^a^	573 ± 51	575 ± 54	<0.00001
**Erythema**				
Male	428 ± 19^a^	425 ± 20	424 ± 20	0.002
Female	408 ± 27	406 ± 20	408 ± 20	0.582
**Individual Typology Angle (ITA, degrees)**				
Male	28.5 ± 18.4	28.2 ± 19.1	27.9 ± 18.8	0.737
Female	44.7 ± 14.7	43.7 ± 14.7	41.2 ± 14.1^a^	0.00004

*Note*: Table entries are the mean ± SD. Site 1 is closest to the wrist and site 5 is closest to the antecubital crease. *p*‐Values are based on a general linear model (GLM) for repeated measures with site as the within repeated measure. Significance of pairwise comparisons between sites are adjusted according to a Bonferroni correction.

^a^ Indicates sites different from the others (*p* < 0.01). At all sites for each parameter, differences between male and female groups was significant (*p* < 0.01).

### 3.3 Variations in skin hydration parameters among sites and between arms

As summarized in Table 4, the TDC measured to a depth of about 2.5 mm (TDC_2.5_) varied among forearm sites on both arms. The most distal forearm site (site 1) tended to have the largest value (33.3 ± 5.5) compared to the most proximal site (site 5) whose average value was 30.9 ± 6.1. For TDC_2.5_, the percentage difference from peripheral to proximal site averaged 7.8%. TDC_0.5_ also tended to be greatest at site 1 (38.0 ± 8.2) compared with site 5 (36.6 ± 8.8) amounting to a 3.8% difference. Although some variation among forearm sites was present, there was no significant difference in either TDC_2.5_ or TDC_0.5_ between arms at corresponding sites. Further analysis revealed that the variation in both TDC_2.5_ and TDC_0.5_ along the forearm is primarily present in female skin and not in male skin as summarized in Table 5. The decreasing TDC values for both TDC_2.5_ and TDC_0.5_ from distal to proximal sites is evident for females and absent in males. At every site, male TDC values were significantly greater than for females (*p* < 0.001). The overall relationship between TDC_2.5_ and TDC_0.5_ is, as anticipated, highly correlated as shown in Figure 3.

**TABLE 4:** Skin hydration and temperature by forearm site and arm for all 30 subjects.

	Site 1	Site 3	Site 5	*p*‐value (overall)
**TDC_2.5_**				
Left Arm	33.3 ± 5.5^a^	31.9 ± 7.0	30.8 ± 6.8	0.00018
Right Arm	33.4 ± 5.6^a^	30.9 ± 5.8	30.9 ± 5.5	0.000003
Arms Combined	33.3 ± 5.5^a^	31.4 ± 6.4	30.9 ± 6.1	<0.000001
**TDC_0.5_**				
Left Arm	37.8 ± 8.2	37.2 ± 9.5	37.0 ± 9.4	0.022
Right Arm	38.3 ± 8.4^a^	37.4 ± 9.3	36.2 ± 8.2	0.011
Arms Combined	38.0 ± 8.2^a^	37.3 ± 9.4	36.6 ± 8.8	0.023
**Skin Temperature (°C)**				
Left Arm	30.7 ± 1.2	30.6 ± 2.1	31.0 ± 1.1	0.294
Right Arm	30.7 ± 1.2	31.0 ± 1.1	31.0 ± 1.0	0.001
Arms Combined	30.7 ± 1.2	30.8 ± 1.7	31.0 ± 1.0	0.095

*Note*: Table entries are the mean ± SD. TDC_2.5_ and TDC_0.5_ are TDC measurements to effective depths of about 2.5 mm and 0.5 mm respectively with values that are dimensionless. *p*‐Values are based on a general linear model (GLM) for repeated measures with site as the within repeated measure. Significance of pairwise comparisons between sites are adjusted according to a Bonferroni correction.

^a^ Indicates sites different from the others (*p* < 0.01). No parameters significantly differed between arms.

**TABLE 5:** Male versus female skin hydration.

	Site 1	Site 3	Site 5	*p*‐value (overall)
**TDC_2.5_**				
Male	36.8 ± 5.4	35.8 ± 6.3	35.8 ± 4.6	0.272
Female	30.3 ± 3.4^a^	27.5 ± 3.1^a^	26.5 ± 3.2^a^	<0.00001
**TDC_0.5_**				
Male	40.5 ± 9.8	42.3 ± 8.9	42.0 ± 8.3	0.092
Female	35.8 ± 5.9^a^	33.0 ± 5.8^a^	31.8 ± 6.0^a^	<0.00001

*Note*: Table entries are the mean ± SD. TDC_2.5_ and TDC_0.5_ are TDC measurements to effective depths of about 2.5 mm and 0.5 mm respectively with values that are dimensionless. Site 1 is closest to the wrist and site 5 is closest to the cubital crease. *p*‐Values are based on a general linear model (GLM) for repeated measures with site as the within repeated measure. Significance of pairwise comparisons between sites are adjusted according to a Bonferroni correction.

^a^ Indicates sites different from the others (*p* < 0.01). At all sites male values of TDC_2.5_ and TDC_0.5_ were greater than for females (*p* < 0.001).

**FIGURE 3:** Relationship between TDC values measured at different depths. TDC values measured to an effective depth of about 2.5 mm (TDC_2.5_) and a depth of about 0.5 mm (TDC_0.5_) at all 180 forearm skin sites. Solid line is the linear regression with the associated equation shown in the figure. The *r* is the Pearson correlation coefficient and *p* is the significance of the correlation. TDC, tissue dielectric constant.

### 3.4 Correlations between skin hydration and skin color parameters

Measurements of tissue hydration via TDC measurements to an effective depth of about 2.5 mm (TDC_2.5_) included both epidermis and dermis and revealed pattern differences between males and females in the skin hydration—color parameter correlation. For males, based on 84 paired measurements (6 sites x 14 male subjects), the average TDC_2.5_ was 36.1 ± 5.4 and was positively correlated with skin erythema (*r* = 0.231, *p* = 0.035). Contrastingly, for females, whose average TDC_25_ was 28.5 ± 3.6 based on 96 paired measurements (6 sites x 16 female subjects), there was a significant TDC_25_ correlation only with skin melanin (*r* = − 0.301, *p* = 0.003). TDC epidermal measurements to a depth of about 0.5 mm (TDC_0.5_) showed a similar disparity between genders. For males, who had an average TDC_0.5_ of 41.6 ± 9.4, the correlation between TDC_0.5_ and erythema remained significant (*r* = 0.385, *p* = 0.001). Similarly, for females, who had an average value of TDC0.5 of 33.5 ± 6.1, the correlation between TDC0.5 and melanin remained as the only significant correlation (*r* = −0.236, *p* = 0.020).

### 3.5 Correlations between Fitzpatrick scores and ITA values

The Fitzpatric classifications have a range between 1 and 6 and were determined by the score obtained from subject responses to the questionairre as described in the methods section. For the male group the scores ranged from 18 to 33 and for the female group from 15 to 35. The ITA value depends on the skin's luminance (L*) and yellow chroma (b*) and was measured at each site with the average ITA of the six measured sites obtained (ITA_AVG_) for each subject. As expected there was a strong positive correlation between the Fitzpatrick score and classification (*r* = 0.909, *p* < 0.001) but there was also a significant negative correlation between the Fitzpatrick score and ITA_AVG_ (*r* = −0.756, *p* < 0.001). This overall relationship shown in Figure 4, was found to be similar for both sexes, with correlations being for females (*r* = −0.687, *p* = 0.003) and for males (*r* = −0.761, *p* = 0.001).

**FIGURE 4:** Relationship between ITA value and Fitzpatrick score. The ITA is shown to be negatively correlated to the FS. The ITA value is determined as the average for all six sites per person. The dotted line is the linear regression with the associated equation shown in the figure. The *r* is the Pearson correlation coefficient and *p* is the significance of the correlation. ITA, individual topology angle; FS, Fitzpatrick score.

## 4 DISCUSSION

The current study offers a comprehensive analysis of skin hydration and color parameters, revealing substantial variances among different sites on the forearm. By including both sexes in the study we were able to observe notable disparities between these aspects with males generally exhibiting higher hydration levels and darker skin tones. These findings are of considerable interest as they provide new insights into the relationship between skin hydration and color.

Our results are consistent with previous studies that have reported sex‐related disparities in skin hydration and color parameters. For example, our findings support previous research by Lubberding et al.^15^ and Mayrovitz et al.^16^ and confirm that males typically display higher hydration levels than females at dermal and epidermal depths. We found a significant correlation between melanin and epidermal hydration in females. These findings align with a negative correlation between L* and stratum corneum hydration observed in Puerto Rican females by Regueira et al.,^27^ further supporting the relationship between darker skin pigmentation and greater water‐retaining capacity. In contrast, other studies found no direct relationship between darker skin color and hydration. However, these studies examined other exposures affecting skin lightness; one study found lower hydration in darker, highly‐UV‐exposed skin, and the other found a lightening (increase in L*) effect of mineral water with increased skin hydration.^18^, ^20^

The higher hydration levels observed in males may be attributed to differences in skin structure and composition, such as thicker dermal layers and higher sebum production.^15^, ^16^ Additionally, the significant correlation between skin hydration values and MI in females suggests that melanin may influence the skin's water‐holding capacity within the dermis, possibly due to its protection against UV radiation,^7^ which can impact skin barrier function and hydration. Furthermore, the variation in melanin and ITA values across different forearm sites suggests that anatomical differences, rather than localized skin exposure, are more relevant due to proximal sites being darker than distal sites of the ventral forearm.

Understanding how skin color affects hydration is important to customize dermatologic treatments and skincare products based on individual skin type and demographic factors. For example, the present study found a link between erythema and increased epidermal hydration in males. This correlation needs further investigation, but it could have clinical implications for conditions like rosacea. Since rosacea has multiple contributing factors, including genetics, immune or neurovascular dysregulation, and environmental factors,^43^ treating it differently in males than in females may be necessary. The relationship between skin hydration, cutaneous blood flow, and erythema needs more evaluation. It might be more beneficial to target the specific cause of erythema in males using vasoconstrictive medications, such as oxymetazoline, instead of addressing other contributing factors.

### 4.1 Study limitations

This study's strengths include comprehensive epidermal and dermal hydration measurement, incorporation of both sexes, and a focus on multiple skin color parameters. However, limitations consist of a relatively small sample size and the specific age range of participants, which may restrict the generalizability of the findings. Additionally, we did not assess other aspects contributing to water retention, such as body composition (fat vs. muscle mass), diet, or water intake. Future studies should involve a larger and more diverse population, assess variables of interest such as body fat percentage, and incorporate longitudinal measurements to assess changes over time. Delving deeper into the underlying mechanisms driving the observed correlations between skin color and hydration includes potentially exploring genetic, hormonal, and environmental influences. Expanding studies to include different anatomical sites and broader age ranges can yield more comprehensive insights into skin hydration and color dynamics. Lastly, investigating the impact of skincare products on these parameters can aid in developing targeted treatments for various skin types and conditions.

## 5 CONCLUSION

This study aimed to explore the relationship between skin hydration and skin color parameters, with a specific focus on gender differences. Our findings revealed substantial correlations between these parameters, indicating that males generally have higher skin hydration levels and greater melanin indices. These results are consistent with previous research and offer new insights into the relationship between skin hydration and color. Notably, the observed correlations, particularly the link between MI and hydration in females, suggest that melanin significantly impacts the skin's water‐holding capacity. These findings hold significance for dermatological assessments and the customization of skincare treatments tailored to individual skin types and demographics.

The study improves our understanding of skin hydration and color dynamics, providing a foundation for future research and clinical applications in personalized skincare and dermatological assessments. Future research should address the limitations of our study, such as the small sample size and specific age range, by expanding the demographic scope and investigating other potential contributing factors. Ultimately, these findings have the potential to provide more efficacious dermatological treatments by focusing on customized approaches to one's gender, skin type, and pathology.

## CONFLICT OF INTEREST STATEMENT

All authors declare no conflicts of interest.

## Data Availability

The data that support the findings of this study are available on request from the corresponding author. The data are not publicly available due to privacy or ethical restrictions.
